# The Role of Stellate Cells in Pancreatic Ductal Adenocarcinoma: Targeting Perspectives

**DOI:** 10.3389/fonc.2020.621937

**Published:** 2021-01-14

**Authors:** Yang Wu, Chun Zhang, Kuirong Jiang, Jens Werner, Alexandr V. Bazhin, Jan G. D’Haese

**Affiliations:** ^1^Department of General, Visceral, and Transplant Surgery, Ludwig-Maximilians-University Munich, Munich, Germany; ^2^Pancreas Center and Pancreas Institute, Nanjing Medical University, Nanjing, China; ^3^German Cancer Consortium (DKTK), Partner Site Munich, Munich, Germany

**Keywords:** pancreatic stellate cells, pancreatic ductal adenocarcinoma, tumor microenvironment, stroma-targeting strategy, tumor therapy

## Abstract

Pancreatic ductal adenocarcinoma (PDAC) is a gastrointestinal malignancy with a dismal clinical outcome. Accumulating evidence suggests that activated pancreatic stellate cells (PSCs), the major producers of extracellular matrix (ECM), drive the severe stromal/desmoplastic reaction in PDAC. Furthermore, the crosstalk among PSCs, pancreatic cancer cells (PCCs) as well as other stroma cells can establish a growth-supportive tumor microenvironment (TME) of PDAC, thereby enhancing tumor growth, metastasis, and chemoresistance *via* various pathways. Recently, targeting stroma has emerged as a promising strategy for PDAC therapy, and several novel strategies have been proposed. The aim of our study is to give a profound review of the role of PSCs in PDAC progression and recent advances in stroma-targeting strategies.

## Introduction

About one century after Karl von Kupffer discovered hepatic stellate cells (HSCs) in 1876, similar star-shaped vitamin A-storing cells (later known as PSCs) in the pancreas were first observed by Wateri et al. in 1982 (1). However, scientists cannot study these cells in both health and pathology until two landmark articles outlined the *in vitro* isolation and culture methods of PSCs in 1998 (2, 3). From then on, emerging studies focused on this new field, and PSCs are now well known as the main cause of the stromal/desmoplastic reaction which is the typical feature of PDAC and chronic pancreatitis (CP) (4–7).

As a malignancy with poor clinical outcomes (8), PDAC develops when pancreatic cells grow out of control and acquire the ability to invade other organs of the body (9, 10). The cancer-centric therapeutics have shown dismal efficacy in eradicating PDAC, since the severe fibrogenic stromal reaction plays both tumor-supporting and -restraining roles in tumor progression and chemotherapy resistance (4, 11–13). As the most abundant stromal cells and major ECM producers, activated PSCs (aPSCs) are known as the critical participants in the stromal/desmoplastic reaction which characterizes PDAC (4). In addition, the dynamic interaction among PSCs, PCCs and other stroma cells create an extremely complex microenvironment which plays a pivotal role in PDAC progression (14, 15). Therefore, PSCs have received great attention, and targeting PSCs has emerged as a hopeful strategy for PDAC therapy recently (12, 14). In this article, we will review the role of PSCs in the development of PDAC and novel therapeutic targets proposed by PSC-related studies.

## PSCs in the PDAC

### Different Phenotypes of PSCs

PSCs can present in two different phenotypes: the quiescent and activated types. In health, PSCs are located in the peri-acinar or interlobular regions of normal pancreas and show a quiescent status (qPSCs), with many perinuclear droplets and a low capacity to produce ECM (2, 3). qPSCs comprise around 4% of the local cells in pancreas (15) and participate in the vitamin A storage, immunity, normal exocrine and endocrine secretion, and the maintenance of normal architecture of the pancreas (16). qPSCs could express desmin, glial fibrillary acidic protein (GFAP), vimentin, nestin, nerve growth factor, and neural cell adhesion molecule (14). Recently, Nielsen et al. indicated that cytoglobin and adipophilin were markers of qPSCs in the normal human pancreas (17).

Numerous mechanisms are involved in the activation process of qPSCs, including risk factors (*e.g.* smoking, alcohol intake, CP), environmental stress (*e.g.* oxidative stress and hypoxia), elevated secretion of factors and signaling pathways (18) (**Figure 1**). During the development of diseases like PDAC or CP, qPSCs can transform into a myofibroblast-like phenotype (19, 20). aPSCs show a positive immunostaining of *α*-smooth muscle actin (*α*SMA), loss of intracellular lipid droplets, enhanced release of numerous molecules, elevated migration and proliferation ability, high ECM protein production [*e.g.* collagens, laminin, hyaluronic acid (HA) and fibronectin] as well as the imbalanced secretion of tissue inhibitors of metalloproteinases (TIMPs) and matrix metalloproteases (MMPs), thus profoundly remodeling TME (19, 20). **Table 1** listed the features of qPSCs and aPSCs.

**Figure 1:** The origin and the activation of PSCs. PSCs are derived from bone marrow, mesenchymal cells and CCR2+ monocytes. qPSCs get activated by several cytokines and transformed into a myofibroblast-phenotype.

**Table 1:** The features of qPSCs and aPSCs.

Features	qPSCs	aPSCs	Pathways in the activation
Vitamin A-rich lipid droplets	Positive	Negative	MAPK (ERK, JNK, p38); Rho/ROCK; NF-*κ*B; PPAR-*γ*; PI3K/Akt; JAK/STAT; Smads; Hedgehog
*α*SMA	Negative	Positive	
Vimentin, GFAP, Desmin	More	Less	
Migration, Proliferation, ECM release abilities	Weak	Strong	
MMPs and TIMPs’ secretion	Normal secretion	Unbalanced secretion of MMPs and TIMPs	
Cytokines, chemokines, growth factors’ production	Low	High	

### Origins of PSCs

The origins of stellate cells are still under investigation. The mesoderm (21–23), neuroectoderm (24, 25) and endoderm (26, 27) were suggested to be the origins of stellate cells. The exact source of PSCs is unclear, since they express a range of neuroectodermal and mesenchymal markers (28). Two *in vivo* studies have suggested that bone marrow is a major source of PSCs (29, 30). Recently, Ino et al. found that C-C chemokine receptor type 2 (CCR2)^+^ monocytes could infiltrate the pancreas *via* the monocyte chemoattractant protein-1 (MCP-1)/CCR2 pathway and differentiate into PSCs (31). However, research on the origins of PSCs is still lacking. Given that PSCs and HSCs exhibited significant similarities through morphological, functional, and gene expression studies (12, 32), research on HSCs will be of reference significance. Cell lineage tracing research demonstrated that HSCs originated from mesenchymal cells and evolved from the mesoderm (23, 33). PSCs might also derive from the neural lineage since they show a positive expression of neuroectodermal markers like GFAP and nerve growth factor (NGF). Similar tracing studies are urgently needed to determine the exact origins of PSCs. Since PSCs are also heterogeneous, a single origin will not derive the entire population but may contribute to the total cell pool what we call PSCs. In-depth understanding of the different origins of PSCs will help us discover their essence and facilitate the development of clinical treatment for PDAC.

### PSCs Heterogeneity and Biomarkers

The heterogeneity of PDAC and PSCs has been widely discussed and studied recently (28, 34). Several distinct cell subgroups with different biomarkers contribute to the heterogeneity of PSCs. Disparate PSCs subsets have multiple functions in PDAC and act as the promoter or preventer in PDAC development.

There have been many studies on the functional heterogeneity of PSC subpopulations with different biomarkers recently. Ikenaga et al. indicated that CD10+ PSCs significantly enhanced the aggressiveness of PCCs compared with CD10− PSCs and were correlated with a poor prognosis of PDAC patients (35). Öhlund et al. reported that PSCs could differentiate into two distinct cancer-associated fibroblasts (CAFs), one (located near tumor cells) expressed higher *α*SMA and exhibited a myofibroblast phenotype, while the other (located more distantly from cancer cells) expressed lower *α*SMA and secreted higher inflammatory factors like interleukin-6 (IL-6), IL-11 (36). The functional heterogeneity of PSCs was also reported by Tjomsland et al. that PSCs from patients showed disparate hepatocyte growth factor (HGF) production which caused distinct cancer outcomes (37). PSC subsets can also exhibit a tumor suppressor effect. CD271+ PSCs were observed around tumor and were significantly correlated with a better prognosis of PDAC patients (38). This further supported the concept that diverse populations of PSCs exhibit disparate or even opposite functions in cancer. In addition, several other biomarkers of PSCs have been reported recently and deserve further research on heterogeneity. S100A4 was discovered as a new biomarker for cancer-derived PSCs (39, 40). Another marker cadherin-11 was found to be upregulated in activated PSCs and was involved in the migration of PCCs (41). Galectin-1 was overexpressed in PSCs and was involved in enhancing the malignancy of cancer cells and forming an immunosuppressive TME of PDAC (42–44). Yoshida et al. demonstrated that kindlin-2 was highly expressed in PSCs and could promote the proliferation and migration of PCCs (45). Higher kindlin-2 expression in stroma was correlated to shorter recurrence-free survival after R0 resection of PDAC (45). More recently, Yeo et al. indicated that p21-activated kinase 1 (PAK1) was expressed in PSCs and could regulate the activation and apoptosis of PSCs. PAK1-knockout mice with PDAC showed an increased survival compared to the control group (46). Biomarkers of PSCs which promote or suppress PDAC were summarized in **Table 2**.

**Table 2:** PSCs biomarkers related to the development of PDAC.

Biomarkers	Description
Cadherin-11	Cadherin-11 is elevated in PSCs and is related to PCCs migration (41).
CD10	CD10^+^ PSCs augment the aggressiveness of PDAC (35).
CD271	CD271^+^ PSCs are around tumor and are associated with a better prognosis of PDAC (38).
Circulating PSCs	PSCs can migrate to metastatic sites together with PCCs *via* circulating blood, which further forms a niche for the metastasis of PDAC (47).
Galectin-1	Galectin-1 is increased in PSCs and increases PCCs invasiveness (42–44).
HGF	PSCs with different HGF production result in the functional heterogeneity (37).
Kindlin-2	Kindlin-2 is overexpressed in PSCs and enhances the proliferation and migration of PCCs (45).
Palladin	Palladin is highly expressed in stroma and promotes invasion of PCCs (48).
P2X7R	P2X7R is correlated with PSCs’ activity and collagen deposition (49).
PAK1	PAK1 is expressed in PSCs and regulate the activation and apoptosis of PSCs (46).
S100A4	S100A4 is a new biomarker in activated PSCs (50).

It is worth noting that, simple inhibition of signaling pathways without considering the heterogeneity of PSCs might cause treatment failure in different PDAC patients. Increasing the identification of PSC biomarkers for different subgroups will not only help gain a better understanding of their heterogeneity and origin but will also facilitate the development of selective therapeutic targeting in PDAC treatment.

## The Role of PSCs in the Aggressiveness of PDAC

The poor prognosis of PDAC is attributed to several reasons, among which the highly desmoplastic TME is the major cause of treatment failure of conventional chemotherapy (51–53). The role of TME in tumor progression has received great attention only in recent decades, although the ‘seed and soil’ theory was first proposed in 1889 (54). The TME of PDAC accounts for up to 90% of tumor volume and contains ECM, PSCs, endothelial cells, collapsed vessels and immune cells (55, 56). Constituting approximately 50% of the TME, activated PSCs have been considered as one of the most significant cell types in PDAC stroma and have received enormous attention in the recent decades (57–69).

The critical roles of PSCs in PDAC aggressiveness include the ECM production, the regulation of desmoplastic reaction, and the modulation of PDAC malignancy in cell proliferation, migration, invasion, angiogenesis, and drug resistance (70). The importance of the crosstalk between PSCs and PCCs in PDAC progression has been well recognized. activated PSCs release increased levels of various cytokines and growth factors, which regulate the proliferation, migration, and invasion of PCCs (14, 18, 71). In addition, PCCs release cytokines like IL-1, IL-6, colony-stimulating factor 1 (CSF1) and tumor necrosis factor-α (TNF-α) and growth factors such as TGF-*β*1 and platelet-derived growth factor BB (PDGF-BB), which modulate the activation of PSCs (13, 72, 73). PSCs also interact with other stroma cells like endothelial cells, immune cells, and neuronal cells, which further contributes to the aggressiveness of PDAC. **Figure 2** is a schematic diagram of PSCs’ activation procedure and the crosstalk of PSCs, PCCs, and other stromal cells in PDAC progression.

**Figure 2:** Schematic diagram of PSC activation procedure and the crosstalk of PSCs, PCCs, and other stromal cells. PCCs induce PSC transformation from a quiescent to an activated state by paracrine stimulation. Activated PSCs release various molecules which in turn promote the aggressiveness of PCCs. In addition, PSCs remain in an activated state showing increased migration, proliferation, and ECM production *via* an autocrine way. PSCs contribute to increased angiogenesis *via* interacting with endothelial cells. PSCs also secrete neurotrophic factors, leading to pain in PDAC. In addition, PSCs play an important role in creating an immunosuppressive TME *via* the crosstalk with immune cells.

### PSCs in Microenvironment Remodeling of PDAC

PDAC is characterized by a severe desmoplastic reaction as well as the energy metabolism disorders (74, 75). As the most prominent cell type in the PDAC-TME, PSCs act an important role in reshaping PDAC-TME both mechanically and metabolically.

#### PSCs in Mechanical Reprogramming of TME

Accumulating evidence reveals that physical factors (*e.g.* tissue pressure, matrix stiffness) are key players with both tumor-supporting and -restraining functions in the development of tumor (76–78). It is well known that PDAC is featured by the rich stroma and severe fibrotic reaction which are attributed to PSC-produced ECM mechanics. The regulation of mechanosensitive ion channels of PSCs, focal adhesion molecules, and cytoskeletal modifications has been shown to act a role in the PSC-mediated mechanobiological remodeling of TME. Fels et al. showed that high interstitial pressure could enhance the activation of PSCs and perpetuate the ECM deposition (79). This positive feedback between activated PSCs and intratumoral pressure could be inhibited by targeting canonical transient receptor potential 1 (TRPC1) (79). Another study showed that the TRPC3 and KCa3.1 channels improved the migration and chemotaxis of PSCs (80). Lachowski et al. revealed that matrix rigidity could directly control the activation and durotaxis in PSCs using a physiomimetic system (81). PSCs were shown to overproduce ECM proteins and induce an aggressive phenotype of PCCs *via* the focal adhesion kinase (FAK)/*β*1 integrin pathway (82). Moreover, the high secretion of ECM also led to the increased interstitial pressure in PDAC (83), which contributed to vascular atrophy, hypoxia, insufficient blood flow, and depletion of nutrients (84). Two recent studies indicated that under hypoxic condition, PSCs exhibited adaptation to oxidative stress and kept continuously activated, increased migration ability, and released elevated molecules like MMP-2, MMP-3 that influenced the ECM remodeling (85, 86). The role of PSCs in remodeling TME mechanically can be further evidenced by the studies using all-trans retinoic acid (ATRA) and tamoxifen. Chronopoulos et al. demonstrated that ATRA could mechanically decrease force-mediated ECM deposition by reducing PSC-produced high traction forces, thereby inhibiting the invasion of PCCs in 3D organotypic models (87). Cortes et al. found that tamoxifen (an agonist of the G protein-coupled estrogen receptor) could inhibit PSC differentiation into myofibroblasts, thereby hampering the PSCs’ ability of remodeling the ECM and enhancing invasion of PCCs (88).

Notably, the mechanically remodeled TME also has an ability of suppressing tumor. Rhim et al. showed that simple depletion of stroma components led to a more aggressive tumor with undifferentiated histology, increased vascularity, and heightened proliferation in PDAC mouse models (89). This is further confirmed by a recent study indicating the tumor-restraining role of activated PSCs and desmoplasia in the high-grade PDAC (13).

In summary, the positive feedback between mechanical TME and activated PSCs is a vital player in the progression of PDAC. Reshaping the TME mechanically by targeting PSCs is a promising approach for the treatment of PDAC. In addition, we need to pay special attention to the suppressing role of PSCs and desmoplasia when formulating tumor treatment strategies, especially in high-grade PDAC.

#### PSCs in Metabolic Remodeling of TME

In addition to the mechanical factors in the microenvironment, the biochemical components also significantly affect cancer. During tumor development, glutamine addiction and cell autophagy play important roles in tumor cell metabolism. PSCs and PCCs present a mutually promoting relationship in cell growth and metabolism. For instance, upregulation of sonic hedgehog (SHH) induced by oncogenic KRAS mutations in PCCs can activate PSCs. Activated PSCs subsequently stimulate the phosphoinositide 3-kinase (PI3K)/protein kinase B (AKT) signaling and respiratory activity in the mitochondria of cancer cells, thereby augmenting oxygen availability for PCCs in the hypoxic TME (90). PDAC has poor blood vessel formation, which creates metabolic stress conditions in PCCs and stromal cells. Su et al. revealed that the metabolic stress could reprogram PSCs, thereby differentially regulating adjacent cells in the TME of PDAC (91). PSC-mediated metabolic remodeling of TME can also support the metabolism of cancer cells even under the nutrient-depleted and hypoxic TME. The “reverse Warburg effect” that indicates the role of stromal cells in maintaining cancer cell metabolism is involved in this process. For example, the autophagy of PSCs can induce alanine production, further fueling the tricarboxylic acid (TCA) cycle, non-essential amino acids (NEAA) and lipid biosynthesis in PCCs (92). In addition, Endo et al. revealed that inhibitors of autophagy could markedly reduce the activation of PSCs as well as tumor invasiveness in PDAC mice (93).

Furthermore, exosomes secreted by PSCs are abundant in cellular metabolites like amino acids and palmitate which fuel the TCA cycle in the nutrient-depleted TME, thereby accelerating the progression of PDAC (94). More recently, Shao et al. found that the positive feedback occurred in Caveolin-1-reactive oxygen species (ROS) signaling in PSCs, leading to a conversion from energy metabolism to glycolysis in PSCs (95). Adjacent PCCs then took up the PSC-produced glycolysis products like lactate to perform oxidative phosphorylation (95). As such, blocking the metabolic coupling between PSCs and PCCs may be a promising treatment for PDAC.

Overall, PSCs are the key players in maintaining the energy metabolism of PCCs *via* autophagy and oxidative stress. More studies are also needed to broaden our understanding and provide novel alternatives to the treatment of PDAC.

### PSCs and Chemoresistance

Recent findings have demonstrated that PSCs play an important role in the chemoresistance of PDAC. PSCs can produce abundant desmoplastic stroma and form a physical barrier preventing the efficacy of chemotherapy drugs, as evidenced by the increased intratumoral drug delivery and penetration after stroma depletion treatment (96–99). Recently, Hessmann et al. found that PSCs showed a drug-scavenging ability by entrapping active gemcitabine (GEM) within the stroma, thus making GEM unavailable for cancer cells (100).

In addition to forming a physical barrier for chemotherapy drugs, PSCs can promote chemoresistance of PDAC by releasing molecules which interact with PCCs (60, 84, 101). For instance, periostin, released by PSCs, was reported to enhance the resistance of PCCs to GEM and promote the invasiveness of PCCs *via* the extracellular signal-regulated kinase 1 and 2 (ERK1/2) and FAK/AKT pathways (102). Singh et al. reported that stromal derived factor-1 (SDF-1) released by PSCs could increase the resistance of PCCs to GEM *via* its receptor C-X-C chemokine receptor type 4 (CXCR4) on cancer cells (103). Additionally, PSC-secreted SDF-1*α* was shown to augment the resistance to GEM *via* ERK1/2 and FAK/AKT pathway in PCCs (104). Amrutkar et al. indicated that PSC-derived fibronectin could induce the drug resistance of PCCs *via* the ERK1/2 pathway (105). Furthermore, Richards et al. showed that exosomes secreted by PSCs caused GEM chemoresistance in cancer cells by transmitting the mRNA of Snail and miR-146a (106). More recently, Xu et al. reported that PSC-secreted HGF increased resistance of PCCs to GEM *via* the c-Met/PI3K/Akt pathway (107).

### PSCs and Metastasis

Accumulating evidence has indicated that PSCs and PSC-derived factors play a critical role in PDAC metastasis. PSCs have been demonstrated to induce the EMT process, a well-known procedure of cancer metastasis initiation, in PCCs (107–109). Kikuta et al. showed that PCCs co-cultured with PSCs attained EMT features like loose cell contacts, a fibroblast-like shape, enhanced migration, decreased epithelial marker expression and increased mesenchymal markers expression (110). Several PSC-released factors are also involved in the induction of EMT in PCCs, such as MMP3 (35), stromal cell-derived factor-1 (SDF-1) (111), vascular endothelial growth factor (VEGF) (112), TGF-*β* (113), connective tissue growth factor (CTGF) (114), periostin (115), HGF (107) and so on. A recent study by Schnittert et al. indicated that PSCs overexpressed integrin *α*11 and increased PDAC metastasis (116). Qian et al. revealed that galectin-1-overexpressed PSCs could enhance the invasion and migration of PCCs by secreting paracrine SDF-1 through the nuclear factor-*κ*B (NF-*κ*B) pathway (43). Apte’s team revealed that PSC-secreted HGF enhanced the aggressiveness of PDAC *via* its receptor c-MET on cancer cells, and HGF inhibition resulted in a significant reduction of metastasis in mouse models of PDAC (117, 118). The investigation by Tian et al. indicated that PCCs could be induced into a more invasive phenotype by the binding of PCC-derived fibroblast growth factor (FGF) to its receptor on PSCs (119). Moreover, a recent research indicated that PSCs overexpressed circRNA hr7:154954255-154998784+ and promoted PDAC metastasis *via* miR-4459/KIAA0513 axis (120).

PSCs can also migrate to metastatic sites together with PCCs, which further forms a niche for the metastasis of PDAC. A hallmark study by Xu et al. indicated that PSCs from the primary tumor area could even be detected and further lead to a severe stromal reaction in the distant metastatic nodules, thereby creating a metastasis-supportive TME (121). Suetsugu et al. found that after splenic injection of PSCs and PCCs, both types of cells were observed in metastatic sites by tracking PSCs expressing green fluorescence protein (GFP) (122). All these findings further support the “seed and soil” theory with regards to cancer metastasis. Therefore, a recent review by Pang et al. recommended to test circulating PSCs together with circulating tumor cells as potential biomarkers in PDAC (47).

### PSCs and Immune Tolerance

PDAC is also characterized by the evasion of host immune surveillance and several studies have indicated that PSCs also play a significant role in this process (42, 123–125).

Ene-Obong et al. demonstrated that PSC-derived SDF-1 showed a chemotactic effect on CD8+ T cells, thereby hampering their infiltration into tumor areas (126). PSCs were also reported to highly secret TGF-*β*1 and IL-10, which had a suppressive effect on dendritic cells (DCs), thus impeding immune responses in PDAC (127). Additionally, two studies suggested that myeloid-derived suppressor cells (MDSCs) were stimulated to differentiate and expand by PSCs *via* IL-6/signal transducer and activator of transcription 3 (STAT-3) signaling pathway and formed a TME resistant to immunotherapy (84, 128). Moreover, research indicated that the level of MDSCs was upregulated in the TME and was related to a poor prognosis (124, 125). The work by Tang et al. revealed that PSC-secreted galectin-1 impeded the activation of T cells, induced their apoptosis and increased the secretion of cytokine by T helper type 2 (Th2), thus forming an immunosuppressive TME of PDAC (42). Lunardi et al. demonstrated that PSC-secreted CXCL10 improved recruitment of CXCR3+ regulatory T cells (Tregs) and reduced cytolysis intermediated by T cells and natural killer (NK) cells, thereby causing the immunosuppressive and tumor-promoting effects (129). PSCs are also involved in the regulation of mast cells as well as mast cell-mediated tumor growth. Ma et al. reported that PSCs activated mast cells which subsequently released IL-13 and tryptase, thus stimulating the proliferation of PCCs and PSCs (130). In addition, PSCs expressed a variety of Toll-like receptors (TLRs) and reacted to TLR ligands, resulting in the activation of signaling pathways and proinflammatory responses (131). Fibroblast activation protein α (FAPα) was reported to interfere antitumor immunity. Kraman et al. revealed that depletion of FAP-α^+^ cells in stroma induced the immune response-mediated tumor regression in a subcutaneous mouse model of PDAC (132).

Overall, PSCs affect the anti-tumor immune by attenuating the viability of immune cells, impairing the immune response as well as augmenting the immune tolerance of PCCs. Recently, immunotherapy has been effective in cancers like melanoma and non-small cell lung cancer, while similar therapies developed for pancreatic cancer have showed little effects. Given that PDAC has a unique immunosuppressive TME, understanding these complex interactions between PSCs and immune cells will help develop more effective immunotherapies against PDAC.

### PSCs and Angiogenesis

In PDAC, PSCs can secret lots of pro-angiogenic factors, such as VEGF, bFGF, IL-8, PDGF, and periostin, which promote proliferation, survival, and migration of endothelia cells, thereby contributing to angiogenesis (133). Tang et al. found that prokineticin (PK) secreted by aPSCs promoted angiogenesis by inducing the function of the PK/PKR system on endothelial cells (133). Kuninty et al. showed that TGF-*β*-activated PSCs induced tube formation (a measure of angiogenesis) of endothelial cells, which could be regulated *via* the therapeutic miRNA-199a-3p and miRNA-214-3p (134). Patel et al. showed that PSCs increased proliferation and tube formation of microvascular endothelial cells *via* the HGF/c-Met pathway (135). In addition, PSCs expressed more type I collagen and VEGF, and showed more pro-angiogenic responses under hypoxia (136). PSCs may have the ability to maintain a balance between pro- and anti-angiogenic responses within PDAC, since PSCs were also reported to release anti-angiogenic molecules like thrombospondin-1 (137), vasohibin-1 and endostatin (138).

Apart from the signaling pathway, PSC-mediated desmoplasia may also affect the vasculature *via* inducing matrix stiffness and ECM deposition. Tissue stiffness is well acknowledged to change cell behaviors (*e.g.* migration, cell–cell adhesion, and proliferation) which are necessary for angiogenesis. For example, Bordeleau et al. revealed that elevated matrix stiffness induced invasion of endothelial cells and neovascular formation by upregulating MMPs in endothelial cells (139). In addition, these alterations in endothelial cells could reduce the barrier function of vessels (139). Similarly, Reid et al. revealed that elevated matrix stiffness upregulated N-cadherin expression on the surface of endothelial cells, thus enhancing the interaction between tumor cells and endothelial cells (140). In addition, the dense stroma can compress the vessels, thereby causing the poor vascularization, nutrient depletion, hypoxia and poor delivery of drugs in PDAC-TME (141). Depletion of PSCs in PDAC led to suppressed angiogenesis, enhanced tumor hypoxia without improving the efficacy of GEM (142). This might be explained by the ECM deposition in the TME covering the local proangiogenic ability of PSCs. Therefore, normalizing, rather than simply depleting the vasculature may be a better strategy to increase the delivery of chemotherapy drugs to tumors.

### PSCs and Nerve Interaction

PSCs are also involved in neural invasion in PDAC progression. Li et al. demonstrated that activated PSCs induced neurite outgrowth towards PCCs and promoted neural invasion of PCCs (143). More recently, Nan et al. reported that PSCs promoted the perineural invasion of PCCs *via* the HGF/c-Met pathway (67). In addition, Han et al. reported that PSCs contributed to pain in PDAC by PSC-induced secretion of pain factors from dorsal root ganglia (144). Demir et al. also found that conditioned medium from cancer-associated PSCs could stimulate neuron outgrowth (145).

## Current Progress in Targeting Strategies

Although the field of PSCs is young, many researchers have engaged great efforts and several strategies targeting the tumor stroma have been proposed (43, 46, 59, 102, 134, 146, 147). However, the strategy of simple PSC depletion was shown to cause more invasive and undifferentiated PDAC with reduced survival in transgenic mice (148). Therefore, most current strategies have focused on normalizing PSCs or reducing ECM production (137, 149–151). In addition, recent research demonstrated that activated PSCs showed a tumor-suppressing function in high-grade PDAC, and normalizing PSCs might be not suitable for this situation (13). The detailed information of current targeted strategies is summarized in **Table 3**. The following paragraphs will mainly focus on the current progress of several promising strategies.

- Vitamin A derivatives: ATRA is a medication used for the treatment of acne and acute promyelocytic leukemia (174, 175). Although several studies have explored the use of ATRA for the treatment of PDAC, there is no solid tumor indication for the drug. Previous experimental studies have indicated that Vitamin A analogs are able to normalize PSCs and induce a less aggressive behavior of PCCs. Chronopoulos et al. indicated that ATRA-treated PSCs significantly decreased the PSC-induced matrix remodeling as well as the invasion of PCCs (87). In KPC mice, ATRA was shown to reprise the quiescent state of PSCs, thereby reducing PCCs proliferation and increasing PCCs apoptosis *via* Wnt-*β*-catenin signaling pathway (176). Single treatment of PCCs with ATRA showed no effects on cancer cell aggressiveness, while drug combination of ATRA and chemotherapy drugs like GEM could markedly decrease tumor growth, epithelial-mesenchymal transition (EMT) as well as modulating several signaling pathways (*e.g.* Wnt, SHH) in KPC mice (177). Furthermore, an in-vivo study showed that after treatment with gold nanoparticles containing ATRA and heat-shock protein 47 siRNA, PSCs got normalized and GEM delivery to the tumor was improved in a mouse model of PDAC (178). All these data provide a sufficient theoretical basis for conducting clinical trials. Recently, a trial (NCT03307148) repurposing ATRA as the stromal targeting agent along with GEM and nab-paclitaxel for PDAC is underway and its phase Ib trial (NCT03307148) has showed that ATRA+GEM+nab-paclitaxel treatment in advanced, unresectable PDAC patients is safe and tolerable (179).
- Vitamin D (VD) analogs: Epidemiological studies have indicated the importance of VD in PDAC progression. Scientists from America and Australia have revealed that the risk and mortality rate of PDAC are negatively related to ultraviolet radiation (UVR), a main source of VD (180–183). More recently, Garland et al. showed that the incidence of PDAC in countries with low UVR is about 6 times that in countries with high UVR, indicating an inverse association between cloud-adjusted UVR and PDAC incidence (184). In addition, the relationship among VD, VD receptor (VDR) and prognosis of PDAC were reported. Investigators demonstrated that low expression of VDR or low circulating VD level (<20 ng/ml) was related to a poor prognosis of PDAC (185–187). Gene expression profiling studies demonstrated that PSCs showed a strong expression of VDR (137). Several studies have showed that VD derivatives could reprise the quiescent state of PSCs and reduce the fibrosis in CP and PDAC (137, 188). Combination therapy of calcipotriol and GEM was shown to reduce the fibrotic reaction in TME and tumor growth, elevate GEM delivery into tumor, and increase survival in KPC mice (137). miR-10a was shown to have a pro-tumorigenic ability (189). Kong et al. found that treatment with VD derivates could markedly inhibit the release of exosomal miR-10a-5p in PSCs, thus reducing its tumorigenic effects on PCCs (190). These data constitute a compelling reason for clinical trials combining VD analogs with chemotherapy in PDAC. Single application of VD derivates seems to be ineffective in PDAC treatment, evidenced by the failure of EB1089 or Arachitol treatment in patients with unresectable PDAC (191, 192). The combination therapy with VD analogs and chemotherapy shows good prospects. Blanke et al. performed a phase II trial evaluating the effects of calcitriol with docetaxel in 25 patients with inoperable PDAC (193). Patients treated with this combination therapy showed an increase in time to progression compared to those received single docetaxel treatment (193). Another phase II study (NCT02754726) was also conducted to evaluate the combination strategy (nivolumab, cisplatin, nab-paclitaxel, paricalcitol, GEM) and the preliminary results were encouraging. The objective response rate in 24 patients was 83%, with a median PFS of 8.17 months and a median overall survival (OS) of 15.3 months (194). Other clinical trials (NCT03472833, NCT03331562, NCT03520790, NCT03300921, NCT03883919, NCT03519308, NCT03415854) are also underway. Taken together, combination strategy of VD analogs and chemotherapy drugs are promising in the treatment of PDAC.
- PEGPH20: Buckway et al. indicated that removal of stromal barrier by hyaluronidase treatment enhanced the penetration of chemotherapy drug in tumor bearing mice (96). PEGPH20, a drug based on the recombinant human hyaluronidase enzyme, was found to reduce the malignant behavior of tumor and promote the survival of mice when combined with GEM in PDAC model (98). Systemic administration of PEGPH20 ablated stromal hyaluronic acid, resulting in increased intratumoral concentration of GEM and an almost doubled overall survival in the KPC mouse model (83). In addition, a phase I trial (NCT01453153) indicated promising results that PDAC patients who were treated with PEGPH20 plus GEM showed prolonged OS and progression-free survival (PFS) rates (99). In another phase II trial (NCT01839487), the largest improvement in PFS was observed in patients with HA-high tumors who received the drug combination (PEGPH20+nab-paclitaxel+GEM) (195).
- SHH inhibitors: It has been well proved that the SHH pathway modulates the interaction between PSCs and PCCs (144). A SHH inhibitor, IPI-926, led to reduced tumor growth and metastasis, increased vascular density and intratumoral GEM concentration in orthotopic mouse models of PDAC (144, 155). Recently, Hwang et al. reported that AZD8542, a novel hedgehog inhibitor, could reduce tumor volume and metastasis in an orthotopic model of PDAC (156). However, an in-vivo study indicated that tumor from SHH-deleted PDAC mice showed a more invasive behavior (161). In addition, the clinical trial of IPI-926 (phase II) was withdrawn because of the increased mortality in PDAC patients (152). The differences between preclinical and clinical setting might attribute to the complicate pathways involved in the stroma-tumor crosstalk. Since every model has its own limitations, any preclinical results should be thoroughly assessed in different models before taken into clinical setting.
- Metformin: Metformin, the first-line medication for the treatment of type II diabetes, is one of the guanidine derivatives from Galega officinalis and is able to decrease the level of blood glucose (196). Research has indicated that metformin shows anticancer effects in several cancers, such as breast, ovarian, pancreatic, and colon cancer (197–199). Duan et al. indicated that metformin suppressed paracrine-mediated activation of PSCs in the coculture setting of PCCs–PSCs (200). Han et al. revealed that metformin inhibited the PSC-mediated desmoplastic reactions, thus reducing tumor size and improving the perfusion of GEM-loaded magnetic nanoparticles in a murine orthotopic PDAC model (157). More recently, metformin was shown to suppress angiogenesis and increase GEM chemosensitivity *via* deactivating PSCs in KPC mice (201). Interestingly, Zechner et al. explored the intratumoral heterogeneity of the therapeutical responses to GEM and metformin in a syngeneic orthotopic mouse model. Metformin was shown to inhibit the proliferation of PCCs close to the desmoplastic part, while GEM reduced the proliferation of PCCs which were away from the fibrotic area, indicating the potential role of PSCs in regulating PCCs sensitivity towards metformin or GEM (200).
- Angiotensin II (Ang-II) inhibitors: It is well acknowledged that the renin-angiotensin system (RAS) plays a role in the activation of PSCs. Ang-II, a key player in RAS, was reported to promote the proliferation and ECM production of PSCs (202). Therefore, the angiotensin blockers are of therapeutic potential and two Ang-II type I receptor inhibitors have been investigated. The work by Masamune et al. demonstrated that Olmesartan reduced the collagen I production of PSCs and impeded tumor growth in PDAC mouse models (163). The other inhibitor, losartan, was also shown to decrease the solid pressure in tumor and increase the vascular perfusion by reducing the collagen and HA production in PDAC mouse models (164).
- Pirfenidone: Pirfenidone is a drug for the treatment of idiopathic pulmonary fibrosis. It has also been shown to reduce PSC activation, collagen secretion, thereby attenuating the proliferation and metastasis of PCCs in a mouse model of PDAC (203). Kozono et al. indicated that compared to treatment with GEM alone, pirfenidone plus GEM could diminish tumor progression by decreasing the activation state of PSCs (203). In another study conducted by Suklabaidya et al., the combination strategy (pirfenidone plus N-acetyl cysteine) diminished the fibrotic reaction, as well as the growth and metastasis of PCCs in a hamster model of PDAC (162).
- CSF1: Since the stroma has the dual effects of promoting and suppressing cancer, simple stroma depletion will bring unpredictable effects in the treatment of PDAC. The circulating level of CSF1 was reported to be elevated in PDAC, and the higher CSF1 level was markedly correlated with more advanced stages of PDAC (204, 205). Recently, a hallmark study by Steins et al. further proved this opinion. They showed that collagens and activated PSCs were lower in the stroma of high-grade mesenchymal PDAC. Further investigation indicated that proliferative and αSMA-positive PSCs had a tumor-restraining effect and high-grade PDAC could deactivate PSCs *via* the secretion of CSF1 (13). Therefore, targeting CSF1 or CSF1R is a promising strategy to maintain a tumor-suppressing TME with abundant collagens and activated PSCs in high-grade PDAC tumors. In addition, the strategy of reprogramming PSCs into a quiescent state should be carefully re-evaluated in high-grade tumor, because it may produce completely different results.
- Some other promising targets: Several other strategies have also been reported recently. For example, the endogenous lipid Lipoxin A4 was demonstrated to impede the activation procedure of PSCs, thereby decreasing the aggressiveness and tumor volume of PDAC *in vivo* (150). Orozco et al. indicated that galectin-1-depleted resulted in the attenuated activation of PSCs, enhanced T cell infiltration, and diminished tumor metastases in mouse models of PDAC (44). Moreover, Yoshida et al. found that calpeptin, a calpain inhibitor, decreased PSC activation and reduced the aggressiveness of PDAC by disrupting the crosstalk between PSCs and PCCs in a mouse xenograft model (159). Yan et al. indicated that exendin-4, a glucagon-like peptide-1 receptor agonist, could inactivate PSCs, thus suppressing PCC proliferation and invasion (167). Xiao et al. reported that resveratrol inhibited hypoxia-induced activation of PSCs, thereby blocking the PSCs–PCCs crosstalk, and decreasing the malignant progression of PDAC and stromal desmoplasia in a KPC mouse model (168). ICG-001, a cAMP-responsive element binding (CREB)-binding protein (CBP)/*β*-catenin antagonist, was shown to suppress the activation of PSCs and PSC-induced migration of PCCs (169). Zhang et al. reported that a heat shock protein 90 (Hsp90) inhibitor, XL888, reduced PSC activation, and enhanced the efficacy of anti-programmed cell death protein 1 (PD-1) blockade in tumor-bearing mice (170). Attempts are also made in reprogramming PSCs by miRNA, a potential therapeutic target (206). Kwon et al. showed that miRNA-29 was reduced in the activation procedure of PSCs, and restoring the expression of miRNA-29 in PSCs decreased the desmoplastic reaction in TME as well as the aggressiveness of PDAC (207). In another study by Asama et al., miRNA let-7d impeded the activation of PSCs by targeting thrombospondin 1, and subsequently decreased pancreatic fibrosis (208). Chen et al. indicated that PSCs treated with nitric oxide could reduce the production of dense stroma, thereby significantly enhancing the efficacy of GEM-loaded liposomes, and inhibiting tumor growth in both subcutaneous and orthotopic tumor mouse models (97). Turaga et al. found that ProAgio specifically depleted PSCs and eliminated angiogenesis, thus increasing drug delivery and GEM efficacy in PDAC (209). Moreover, a study by German cancer research center showed that date palm fruit extracts could reduce PSC-induced fibrosis, decrease PSCs proliferation, and reverse the fibrotic phenotype of PSCs, thereby possibly enhancing the efficacy of known chemotherapy drugs (210).

**Table 3:** Strategies targeting PSCs in TME of PDAC.

Strategies	Descriptions	Main results
Clinical studies		
PEGPH20	HA degradation	Phase Ib: Elevated OS and PFS in PDAC patients (99).
IPI-926	Hedgehog pathway inhibitor	Phase II: Withdrawn for increased mortality (152).
Marimastat	MMP inhibitor	Phase II: No extra benefits were found in PDAC patients, compared to GEM alone (153).
ATRA	Retinoic acid derivatives	Phase Ib: Ongoing, no results released (154).
Cabiralizumab plus nivolumab	Target CSF1R	Phase Ia/Ib: no results published. NCT04191421
Vitamin D3	Target VDR	Phase III: no results published. NCT03472833, NCT03300921
Paricalcitol	Target VDR	Phase II: no results published. NCT02754726
Preclinical studies		
IPI-926	Hedgehog pathway inhibitor	Elevated vascular density and concentration of GEM in tumor of KPC mice (155).
AZD8542	Hedgehog pathway inhibitor	Reduced tumor volume and metastasis in an orthotopic model of PDAC (156).
Metformin	Repurposed anti-diabetic drugs	Reduced PSC activation, tumor volume and increased GEM efficacy in an orthotopic mice of PDAC (157).
Minnelide	TGF*β* signaling inhibitor	Reduced ECM production, increased vasculature, improved drug delivery in tumor in both spontaneous KPC mice and PDAC xenografts mice (158).
Calpeptin	Calpains inhibitor	Reduced PSC activation, decreased fibrosis, tumor volume in PDAC xenografts mice (159).
JQ1 & I-BET151	BET inhibitors	Attenuated PSC activation and collagen I production in the mouse model of PDAC (160).
Genetical deletion of αSMA+ cells	αSMA+ cells	More aggressive tumors, increased hypoxia and EMT, reduced survival in transgenic PDAC mice (148).
Genetical deletion of SHH	SHH pathway	Undifferentiated malignancies, increased vascularity and proliferation in SHH-deleted PDAC mice (161).
PEGPH20	HA degradation	Depleted HA, expanded blood vessels and increased chemotherapeutic drug delivery in tumor of PDAC mice (83).
Pirfenidone	TGF*β* signaling inhibitor	Reduced PSC proliferation, collagen production; co-treatment with GEM reduced tumor growth and hepatic metastasis in PDAC mice (162).
Olmesartan	Ang II receptor 1 antagonists	Decreased PSC proliferation, αSMA expression, collagen I production, tumor growth in subcutaneous PDAC mice (163).
Losartan	Ang II receptor 1 antagonists	Decreased stress in solid tumors, improved vascular perfusion, increased chemotherapeutic delivery in PDAC mice (164).
ATRA	Retinoic acid derivatives	Decreased PSC migration, collagen synthesis, leading to an increased apoptosis of surrounding PSCs (151).
Calcipotriol	Vitamin D3 derivatives	Improved intratumoral concentration of drug, decreased tumor size, prolonged survival compared to GEM alone in KPC mice (137).
LXA4	An endogenous bioactive lipid	Reduced PSC activation, fibrosis and tumor growth of in mouse model (150).
Fasudil	Rho-associated protein kinase inhibitor	Reduced PSC activation, decreased collagen deposition, increased GEM delivery, improved OS in PDAC mouse model (146).
AZ13381758	CXCR2 inhibitor	Reduced collagen I/III, lowered metastasis, increased OS in PDAC mouse model (165).
AV3	Integrin α5 inhibitor	Reduced desmoplasia, decompressed blood vasculature, improved GEM efficacy in patient-derived xenograft PDAC model (62).
AMD3100	CXCR4 antagonist	Increased T cell infiltration, reduced tumor growth in PDAC mouse model (166).
AMG102	HGF inhibitor	Reduced tumor volume and metastasis when treated together with GEM in orthotopic mice of PDAC (117).
CSF1	Strong inducer of PSC deactivation	In mesenchymal PDAC, CSF1 deactivated PSCs thereby reducing the tumor-restraining effect of PSCs.
Exendin-4	Glucagon-like peptide-1 receptor agonist	Decreased PSC proliferation and migration, reduced PCC migration, invasion and proliferation (167).
Resveratrol	Natural polyphenol with antioxidant and anticancer effects	Inhibited hypoxia-induced PSC activation, blocked PSCs–PCCs crosstalk, and decreased malignant progression of PDAC and stromal desmoplasia in a KPC mouse model (168).
ICG-001	*β*-catenin/CBP inhibitor	Suppressed activation of PSCs and PSC-induced migration of PCCs (169).
XL888	Hsp90 inhibitor	Reduced PSC activation and enhanced the efficacy of anti-PD-1 blockade in tumor bearing mice (170).
Curcumin	Turmeric polyphenol derivates of rhizomes of Curcuma longa	Reduced *α*SMA, type I collagen, and fibronectin and diminished PSC activation (171).
Emodin	Important component of Aloe vera	Reduced expression of αSMA, type I collagen, and fibronectin in PSCs and enhanced the efficacy of chemotherapeutic drugs for PDAC (172).
Pantoprazole	Proton pump inhibitor	Decreased collagen secretion from PSCs and proliferation of PCCs (173).

## Challenges

It can be clearly seen from the above that, the role of PSCs in PDAC progression and the stroma-targeted strategies have been well acknowledged. Nevertheless, it must be admitted that little benefit has been observed so far in the clinical trials. PSC-targeted strategy has also met several challenges which need to be overcome in the future.

Recently, PSCs have been reported to be heterogeneous, and the heterogeneity of PSCs has received great attention. Ikenaga et al. reported that CD10^+^ PSCs were more effective than CD10^-^ PSCs in inducing invasion and proliferation of PCCs (35). Another research demonstrated two distinct PSCs: a) one subtype expressed high αSMA and displayed a myofibroblast phenotype; b) another subtype showed lower αSMA expression and instead released higher IL-6 and other chemokines (36). As such, different PSC subtypes may have completely distinct effects on PDAC development, and this heterogeneity needs to be carefully considered in the development of novel stroma targeting strategies in PDAC. More research on PSC subtypes is needed to further progress this field.

The complexity of pathways mediating PSCs–PCCs crosstalk is another challenge, although several candidate pathways were reported to be potential targets for novel therapeutic strategies. For example, the clinical trial of IPI-926 (a hedgehog inhibitor) was terminated due to increased mortality of patients (152), though it worked well in pre-clinical experiments (144, 155). Therefore, when testing new therapeutic approaches, it is critical to replicate as much as possible the conditions (*e.g.* hypoxia) inside human pancreatic malignancy. Hopefully, many new research models have been developed recently. For instance, Boj et al. developed organoid models of PDAC which realized heterogeneity, 3D structure, and crosstalk between different cell types (211). Finally, new therapies need to be thoroughly evaluated in different models before we take them into clinical, since each model has its own limitations.

Although most strategies have focused on deactivating PSCs or stroma, the tumor-restraining role of PSCs in PDAC should be carefully considered when designing novel strategies. This is confirmed by the failure of simple stroma depletion strategy. In addition, a recent study further proved the importance of PSCs and stroma in suppressing high-grade mesenchymal PDAC (13). The failure of several PSCs/stroma-targeting studies is likely due to the neglect of the tumor-restrictive properties of PSCs/stroma. Therefore, the strategy of reprogramming PSCs into a quiescent state should be carefully re-evaluated especially in high-grade PDAC.

## Conclusion

As we demonstrated in this review, PSC-produced collagenous stroma is recognized as a major factor of aggressiveness and chemoresistance in PDAC. The crosstalk among PSCs, PCCs, and other stromal cells also plays a key role in immune tolerance, chemoresistance, angiogenesis, metastasis, and recurrence of PDAC. Modulating PSCs can reprogram the cancer ‘soil’ into a tumor-suppressive niche, thereby turning foes into friends that suppress PDAC progression. Additionally, since the standard chemotherapy targeting cancer cells alone has displayed disappointing outcomes, novel stroma-targeting strategies together with conventional chemotherapy has become the research hotspot and various strategies have been proposed. Nevertheless, these therapeutic strategies need to be further validated in appropriate, clinically relevant pre-clinical models before they are assessed in clinic. Hopefully, many preclinical studies demonstrate that normalization of PSCs and PSC-derived ECM can reprogram the stroma into a less tumor-supportive phenotype which further decreases the aggressiveness of PDAC. Several clinical trials are underway and will finally determine the viability and efficacy of these therapeutic approaches against PDAC. Notably, given the tumor-restraining ability of PSCs and stroma, the strategy of deactivating PSCs might cause negative effects and should be carefully re-evaluated in high-grade PDAC. More research is also needed to deepen the understanding of the dual role of PSCs in the development of PDAC.

## Author Contributions

Investigation and writing—original paper, YW and CZ. Equal contribution; writing—review and editing, all authors. Supervision, AB, KJ, and JW. Project administration, AB and JD’H. All authors have read and agreed to the published version of the manuscript. All authors contributed to the article and approved the submitted version.

## Funding

This research has been supported by the Chinese Scholarship Council to YW (201708320343) and to CZ (201708320342).

## Conflict of Interest

The authors declare that the research was conducted in the absence of any commercial or financial relationships that could be construed as a potential conflict of interest.
